The article "Identification of Key Genes and Pathways in Osteosarcoma by Bioinformatics Analysis" was published in 2022. Journal: Comput Math Methods Med.

# Identification of Key Genes and Pathways in Osteosarcoma by Bioinformatics Analysis

**DOI:** 10.1155/2022/7549894

**Published:** 2022-01-15

**Authors:** Xiujin Chen, Nan Zhang, Yuanyuan Zheng, Zhichao Tong, Tuanmin Yang, Xin Kang, Yan He, Liang Dong

**Affiliations:** ^1^Department of Orthopaedic Oncology, Hong Hui Hospital of Xi'an Jiaotong University, Xi'an, 710054 Shaanxi Province, China; ^2^Department of Pathology, Hong Hui Hospital of Xi'an Jiaotong University, Xi'an, 710054 Shaanxi Province, China; ^3^Geriatric Cardiovascular Department, The Second Affiliated Hospital of Xi'an Jiaotong University (Xibei Hospital), Xi'an, Shaanxi Province, China; ^4^Department of Sports Medicine, Hong Hui Hospital of Xi'an Jiaotong University, Xi'an, 710054 Shaanxi Province, China; ^5^Department of Magnetic Resonance Imaging, Hong Hui Hospital of Xi'an Jiaotong University, Xi'an, 710054 Shaanxi Province, China; ^6^Department of Cervical Spine Surgery, Hong Hui Hospital of Xi'an Jiaotong University, Xi'an, 710054 Shaanxi Province, China

## Abstract

**Purpose:**

Osteosarcoma (OS) is the most primary bone malignant tumor in adolescents. Although the treatment of OS has made great progress, patients' prognosis remains poor due to tumor invasion and metastasis.

**Materials and Methods:**

We downloaded the expression profile GSE12865 from the Gene Expression Omnibus database. We screened differential expressed genes (DEGs) by making use of the R limma software package. Based on Gene Ontology, Kyoto Encyclopedia of Genes and Genomes, and Gene Set Enrichment Analysis, we performed the function and pathway enrichment analyses. Then, we constructed a Protein-Protein Interaction network and screened hub genes through the Search Tool for the Retrieval of Interacting Genes.

**Result:**

By analyzing the gene expression profile GSE12865, we obtained 703 OS-related DEGs, which contained 166 genes upregulated and 537 genes downregulated. The DEGs were primarily abundant in ribosome, cell adhesion molecules, ubiquitin-ubiquitin ligase activity, and p53 signaling pathway. The hub genes of OS were KDR, CDH5, CD34, CDC42, RBX1, POLR2C, PPP2CA, and RPS2 through PPI network analysis. Finally, GSEA analysis showed that cell adhesion molecules, chemokine signal pathway, transendothelial migration, and focal adhesion were associated with OS.

**Conclusion:**

In this study, through analyzing microarray technology and bioinformatics analysis, the hub genes and pathways about OS are identified, and the new molecular mechanism of OS is clarified.

## 1. Background

Osteosarcoma (OS) is a common malignant bone tumor and often occurs in children or adolescents under 20 years old. As the most common bone malignant tumor in children, it accounts for about 5% of pediatric tumors [1, 2]. The incidence of OS is 0.20-0.35 per 100,000 people. OS is also associated with high mortality. The 5-year overall survival rate for the primary nonmetastatic OS is 75-77%, and the 5-year survival rate for metastatic OS does not exceed 20% [3]. The pathogenesis of OS includes genetic factors and environmental factors [4]. Currently, the treatment of OS is mainly surgical resection in combination with radiotherapy and chemotherapy. It is helpful for the long-term survival of OS [5]. Nevertheless, despite advances in cancer treatment, the median survival rate of OS is still very low. The recurrence and metastasis rate of OS is high, and the prognosis is poor due to unclear pathogenesis [6]. Therefore, we need more efforts at further clarifying the molecular mechanisms of tumor occurrence and development, which may be beneficial to finding better molecular targets for the cure of OS.

The article "Identification of Key Genes and Pathways in Osteosarcoma by Bioinformatics Analysis" was published in 2022. Journal: Comput Math Methods Med.

Gene expression profile means constructing a cDNA library of cells or tissues in a specific state, which is non-biased [7]. Through large-scale cDNA sequencing, making qualitative and quantitative analysis on the composition of its mRNA population and collecting sequence fragments of cDNA, it is aimed at describing abundant information and gene expression type of specific cell or tissue in a specific state. Wang et al. find through gene expression profile and experimental analyses that lncRNA-CIR can slow down the invasion, proliferation, and migration of OS cells; provide the treatment of OS with a new target; and facilitate OS cell apoptosis [8]. After analyzing the gene expression profile, Fan et al. conclude that CTPS2, TP53I3, and SLC1A1 may have a paramount function on the metastasis of OS. hsa-miR-194, hsa-miR-422a, mmp3, and VEGFB may also take part in the metastasis of OS [9]. Currently, most tumors are classified based on morphology [10]. We urgently need to identify biomarkers to determine tumor subtypes, which may have an impact on prognosis and treatment. We can identify the molecular characteristics of individual patient tumors through making use of gene expression microarrays (GEM) [11] in combination with bioinformatics analysis, and simple hierarchical clustering has resulted in the identification of new cancer categories that transcend the distinction based on immunohistochemistry and morphology.

In this research, we utilize microarray technology and bioinformatics aiming at processing the gene expression profile GSE12865 (gene expression of human pediatric OS tumor samples relative to normal human osteoblasts). Finally, the hub genes and signal pathways related to OS are obtained, which is of great significance for exploring the pathogenesis and searching for biomarkers and treatment methods of OS.

The article "Identification of Key Genes and Pathways in Osteosarcoma by Bioinformatics Analysis" was published in 2022. Journal: Comput Math Methods Med.

## 2. Material and Methods

### 2.1. Acquisition of Microarray Data

As a public functional genomics data repository supporting MIAME-compliant data submissions, Gene Expression Omnibus (GEO) [12] database (https://www.ncbi.nlm.nih.gov/geo) is one of the databases of NCBI (https://pubmed.ncbi.nlm.nih.gov/). GEO accepted array- and sequence-based data aiming at offering tools and helping users query, and download curated gene expression profiles. We observed GSE12865 from the GEO database, and Affymetrix Human Gene 1.0 ST Array was the platform for GSE12865. GSE12865 performed a genome-wide comparison of gene expression in OS tumor tissues relative to normal human osteoblasts (Hob) and identified the differentiated expression genes.

### 2.2. Identification of Differentially Expressed Genes (DEGs)

Through making use of several packages of R statistical software [13] (version 3.3.2, https://www.r-project.org/), we finished the significance analysis of the raw data. When a *P* value < 0.00001 had statistical significance, genes at this threshold were screened as DEGs. Meanwhile, if fold change was >1, it was classified as upregulated DEGs; if fold change was <1, it was classified as downregulated DEGs.

### 2.3. Kyoto Encyclopedia of Genes and Genomes (KEGG) and Gene Ontology (GO) Pathway Enrichment Analysis of DEGs

We performed GO term enrichment analysis and dug out DEG functions and biological significance through making use of the Database for Annotation, Visualization and Integrated Discovery (DAVID; https://david.ncifcrf.gov/tools.jsp).We performed KEGG pathway enrichment analysis aiming at finding pathways in close relation to OS and biological information. We considered *P* value < 0.05 to have statistical significance.

### 2.4. Module Analysis of Protein-Protein Interaction (PPI) Network

We obtained DEG's PPI information by making use of the Search Tool for the Retrieval of Interacting Genes (STRING) database (https://string-db.org). We visualized the PPI network based on PPI information through making use of Cytoscape software [14]. We selected the DEGs which in the PPI network had high connectivity. The higher the degree of connectivity, the closer the connection between DEGs and OS.

### 2.5. Gene Set Enrichment Analysis (GSEA) on the Whole Gene Expression Level

GSEA [15] is a gene set-based enrichment analysis method. When analyzing gene expression data, we first determined the purpose of the analysis and selected one or more functional gene sets for analysis. Sample data files and chip expression configuration files were created and imported into the GSEA software. We selected the corresponding chip platform and gene set database and set other parameter defaults, then, GSEA could be run on the total gene expression level, and the pathway enrichment results could be obtained.

The article "Identification of Key Genes and Pathways in Osteosarcoma by Bioinformatics Analysis" was published in 2022. Journal: Comput Math Methods Med.

## 3. Result

### 3.1. Identification of DEGs

The OS-related gene expression data set GSE12865 included 12 human OS tumor samples and 2 normal human osteoblasts samples. We selected the R language software for the preprocessing of microarray data. When *P* was <0.00001 and the fold change was >1, the gene was upregulated DEGs; when *P* was <0.00001 and the fold change was <1, the threshold gene was downregulated DEGs. A heat map demonstrated expression profiling of DEGs (Figure 1). Significance analysis found that compared with normal samples, there were 703 DEGs in the OS sample, of which 166 DEGs were obviously upregulated and 537 DGEs were obviously downregulated. Top 10 upregulated DEGs included A2M, GUCY1A3, GIMAP4, FLT1, RASGRP3, GIMAP7, CALCRL, HLA-DRA, EMCN, and PTPRB. Top 10 downregulated DEGs included ANGPTL5, NLGN1, MOXD1, FGF5, SLC14A1, PDE1A, MFAP5, CPA4, PTX3, and NPR3.

### 3.2. GO and KEGG Enrichment Analysis of Upregulated DEGs

Based on GO term enrichment analysis, it demonstrated that there were significant differences among the 166 upregulated DEGs enriched in molecular function (MF), biological process (BP) and cellular components (CC). The top 10 enriched BP terms of upregulated DEGs were positive regulation of vasculogenesis, negative regulation of endothelial cell proliferation, sprouting angiogenesis, endothelial cell migration, cell communication and signaling, cardiac ventricle development, cellular response to vascular endothelial growth factor stimulus, regulation of endothelial cell migration, and enzyme-linked receptor protein signaling pathway (Figure 2(a)). Regarding CC, these DEGs were obviously abundant in MHC class II protein complex, MHC protein complex, an integral component of lumenal side of endoplasmic reticulum membrane, late endosome membrane, clathrin-coated endocytic vesicle, clathrin-coated endocytic vesicle membrane, ER to Golgi transport vesicle membrane, lytic vacuole, lysosome, and integral component of the plasma membrane (Figure 2(b)). For MF, these DEGs were obviously abundant in vascular endothelial growth factor-activated receptor activity, transmembrane receptor protein phosphatase activity, transmembrane receptor protein tyrosine phosphatase activity, MHC class II receptor activity, mitogen-activated protein kinase binding, MHC class II protein complex binding, transmembrane receptor protein tyrosine kinase activity, transmembrane receptor protein kinase activity, MAP kinase kinase kinase activity, and protein tyrosine kinase activity (Figure 2(c)). On the basis of KEGG pathway analysis, it demonstrated that the 10 most significant enrichment pathways of upregulated DEGs were allograft rejection, asthma, type I diabetes mellitus, graft-versus-host disease, inflammatory bowel disease, Th1 and Th2 cell differentiation, antigen processing and presentation, hematopoietic cell lineage, cell adhesion molecules, and rheumatoid arthritis (Figure 2(d)).

The article "Identification of Key Genes and Pathways in Osteosarcoma by Bioinformatics Analysis" was published in 2022. Journal: Comput Math Methods Med.

### 3.3. GO and KEGG Enrichment Analysis of Downregulated DEGs

On the basis of the GO term enrichment analysis, it demonstrated that there were obvious significant differences among the 537 downregulated DEGs abundant in BP, MF, and CC. Regarding BP, downregulated DEGs were abundant in mitochondrial translational termination, translational termination, mitochondrial translation, mitochondrial translational elongation, translational elongation, posttranslational protein modification, neutrophil degranulation and activation, neutrophil-mediated immunity taking part in immune response, and cellular protein metabolic process (Figure 3(a)). Regarding CC, downregulated DEGs were obviously abundant in Swr1 complex, mitochondrial large ribosomal subunit, ficolin-1-rich granule lumen, cytoplasmic vesicle lumen, ficolin-1-rich granule, secretory granule lumen, mitochondrial inner membrane, focal adhesion, nucleolus, and mitochondrion (Figure 3(b)). Regarding MF, downregulated DEGs were mainly abundant in insulin-like growth factor II binding, intramolecular transferase activity, guanyl ribonucleotide binding, phosphotransferases, RNA polymerase II activity, insulin-like growth factor I binding, guanyl ribonucleotide binding, ubiquitin-ubiquitin ligase activity, insulin-like growth factor binding, integrin binding, purine ribonucleoside binding, and RNA binding (Figure 3(c)). On the basis of KEGG pathway analysis, it demonstrated that the 10 most significant enrichment pathways of downregulated DEGs were thyroid cancer, citrate cycle (TCA cycle), p53 signaling pathway, tyrosine metabolism, melanoma, bacterial invasion of epithelial cells, TGF-beta signaling pathway, ribosome, Huntington's disease, and human papillomavirus infection (Figure 3(d)).

### 3.4. Analysis of Upregulated PPI Network

Through the STRING database, we acquired related PPI information. The PPI network of 166 upregulated DEGs contains 151 nodes and 106 edges (Figure 4). The top 4 DEGs were selected as hub genes whose connectivity degrees were larger than 10. The degree of KDR was 12, the degree of CDH5 was 11, and the degrees of CD34 and CDC42 were both 10. And the expression levels of KDR, CDH5, CD34, and CDC42 in human OS tumor samples were significantly higher than those in normal human osteoblasts (Figures 5(a)–5(d)).

The article "Identification of Key Genes and Pathways in Osteosarcoma by Bioinformatics Analysis" was published in 2022. Journal: Comput Math Methods Med.

### 3.5. Analysis of Downregulated PPI Network

Through the STRING database, we acquired pertinent PPI information. The PPI network of 537 downregulated DEGs contained 523 nodes and 774 edges (Figure 6). The top 4 DEGs were selected as hub genes whose connectivity degrees were larger than 23. The degree of RBX1 was 26, the degree of POLR2C was 26, the degree of PPP2CA was 25, and the degree of RPS2 was 23. Figures 7(a)–7(d) show the expression levels of RBX1, POLR2C, PPP2CA, and RPS2 in human OS tumor and normal human osteoblasts samples.

### 3.6. GSEA Analysis on the Whole Gene Expression Level

Figure 8 shows the four significantly enriched pathways related to OS, which were cell adhesion molecules (CAMs) (Figure 8(a)), chemokine signal pathway (Figure 8(b)), transendothelial migration (Figure 8(c)), and focal adhesion (Figure 8(d)). These findings suggested new molecular mechanisms when OS occurred and progressed.

## 4. Discussion

As a subgroup of cells, mesenchymal stem cells (MSCs) of the bone marrow stroma are found in mammalian bone marrow stroma that has the potential to differentiate into the bone, cartilage, fat, nerve, and myoblasts [16]. The pathogenesis of OS may be related to the changes in the differentiation pathway of MSCs in mature osteoblasts [17]. The abnormal expression of oncogenes and tumor suppressor genes caused by genetic and epigenetic events deregulates important cell signaling pathways, which also promotes the conditions for the formation of OS [18]. Microarray technology is an emerging molecular biology technique in recent years [19]. It is of great significance for humans to explore the mysteries of life, reveal the nature of diseases, and realize the human genome project [20]. This method uses a manipulator to accurately spot a large amount of DNA on a glass slide. The researchers then label the DNA extracted from the cells they study with fluorescent labels. The labeled probe can be complementary to the DNA on the slide. Then, the slide is placed under the scanner and measure the brightness of each fluorescent spot. The brightness reflects the amount of specific DNA fragments. We analyzed the gene expression profile GSE12865 related to OS by microarray technology and obtained 703 DEGs in total, which were inclusive of 166 genes upregulated and 537 genes downregulated.

GO and KEGG enrichment analyses demonstrated that DEGs were obviously abundant in the ribosome, cell adhesion molecules, ubiquitin-ubiquitin ligase activity, and p53 signaling pathway. The mammalian ribosome is composed of 40 subunits and 60 subunits and requires the coordinated assembly of about 80 ribosomal proteins and 4 different ribosomal RNAs (rRNAs) [21]. Luo et al. find that probably through translational control, ribosomal protein L34 which is expressed highly indicates poor prognosis in OS and its knockdown suppresses OS proliferation [22]. Chong et al. reported that through targeting L1 cell adhesion molecules (CAMs), miR-503 serves as a tumor suppressor in OS [23]. Weisberg et al. found that the CBL mutation of E3 ubiquitin ligase finds in several myeloid tumors caused a decrease in ubiquitin ligase activity [24]. Deng et al. found that the histone deacetylase inhibitor promotes OS cell apoptosis through activation of the p53 signaling pathway [25].

The article "Identification of Key Genes and Pathways in Osteosarcoma by Bioinformatics Analysis" was published in 2022. Journal: Comput Math Methods Med.

The hub genes of OS were KDR (Kinase Insert Domain Receptor), CDH5 (cadherin 5), CD34 (CD34 molecule), CDC42 (cell division cycle 42), RBX1 (ring-box 1), POLR2C (RNA polymerase II subunit C), PPP2CA (Protein Phosphatase 2 Catalytic Subunit Alpha), and RPS2 (Ribosomal Protein S2). KDR-associated diseases are inclusive of hemangioma and capillary infantile, and its related pathways are proteoglycans in cancer and Notch-mediated HES/HEY network [26]. CDH5 is closely related to OS and periapical granuloma, and its pertinent pathways include signal transduction, blood-brain barrier, and immune cell migration [27]. As for PPP2CA, it is in association with neurodevelopmental disorder and language delay with or without structural brain abnormalities and Alzheimer's disease [28]. Pathways in relation to it are S37 mutants of beta-catenin and phosphorylated RET signaling. GO annotations in relation to this gene contain hydrolase activity and protein C-terminus binding. Finally, it is reported that RPS2 is inclusive of retinitis pigmentosa and heart valve dysplasia [29].

GSEA analysis demonstrated the genes of OS are most abundant in cell adhesion molecules, chemokine signal pathway, transendothelial migration, and focal adhesion. Liu and others believe that chemokine receptors and chemokines not only take part in the development of tissue differentiation, inflammation, hematopoiesis, and immune regulation but also have a paramount function when tumors occur and develop [30]. Chemokines are in close relation to the formation and development of tumors.

## 5. Conclusion

We process the gene expression profile GSE12865 (gene expression of human OS tumor samples relative to normal human osteoblasts) by making use of microarray technology and bioinformatics. Finally, we find 703 DEGs, which consist of 166 DEGs upregulated and 537 DEGs downregulated. The pathways of DEGs are primarily abundant in ribosome, cell adhesion molecules, ubiquitin-ubiquitin ligase activity, and p53 signaling pathway. The hub genes of OS are KDR, CDH5, CD34, CDC42, RBX1, POLR2C, PPP2CA, and RPS2. The hub genes and signal pathways related to OS are obtained, which is of great significance for exploring the pathogenesis and searching for biomarkers and treatment methods for OS.

The article "Identification of Key Genes and Pathways in Osteosarcoma by Bioinformatics Analysis" was published in 2022. Journal: Comput Math Methods Med.

## Figures and Tables

**Figure 1:** Cluster analysis heat map of DEGs. The bottom axis stands for samples, the top axis stands for sample clusters, and the left-hand axis stands for DEG clusters. Red refers to upregulated DEGs, and blue refers to downregulated DEGs.

**Figure 2:** GO terms and KEGG enrichment analyses of upregulated DEGs in OS. (a–c) Upregulated DEG enrichment analysis results of BP, CC, and MF. (d) 10 KEGG pathways in which upregulated DEGs were abundant.

**Figure 3:** GO terms and KEGG enrichment analyses of downregulated DEGs in OS. (a–c) Downregulated DEG enrichment analysis results of BP, CC, and MF. (d) 10 KEGG pathways in which downregulated DEGs were abundant.

**Figure 4:** PPI network for DEGs upregulated, which is inclusive of 151 nodes and 106 edges. Nodes mean proteins, and edges mean the interaction of proteins.

**Figure 5:** The expression level of hub genes (a) KDR, (b) CDH5, (c) CDC42, and (d) CD34 in human OS tumor samples and normal human osteoblasts based on GSE12865.

**Figure 6:** PPI network for DEGs downregulated, which contains 523 nodes and 774 edges. Nodes mean proteins, and edges mean the interaction of proteins.

**Figure 7:** The expression level of hub genes (a) RBX1, (b) POLR2C, (c) PPP2CA, and (d) RPS2 in human OS tumor samples and normal human osteoblasts based on GSE12865.

**Figure 8:** The four enrichment plots from the GSEA results. The gene sets of (a) cell adhesion molecules (CAMs), (b) chemokine signal pathway, (c) transendothelial migration, and (d) focal adhesion were significantly enriched in human OS tumor samples based on GSE12865.

## Data Availability

The datasets used and/or analyzed during the current study are available from the corresponding author on reasonable request.
